# TAOK1 Promotes Proliferation and Invasion of Non-Small-Cell Lung Cancer Cells by Inhibition of WWC1

**DOI:** 10.1155/2022/3157448

**Published:** 2022-09-15

**Authors:** Lian Chen

**Affiliations:** Department of Respiratory and Critical Care Medicine, The First Affiliated Hospital of Fujian Medical University, Fuzhou, Fujian 350000, China

## Abstract

**Background:**

For patients with advanced non-small-cell lung cancer (NSCLC), targeted therapy significantly improves the therapeutic effect of NSCLC patients. With the development of molecular targeted therapy, more and more NSCLC-related genes have been found. Thousand and one amino-acid kinase 1 (TAOK1) has been identified as a potential target for drug research in various cancers. The main objective of this study was to explore the expression and function of TAOK1 in NSCLC.

**Methods:**

Western blotting was employed to assess TAOK1 expression in NSCLC cell lines. The effects of TAOK1 on biological behaviors, including proliferation, invasion, and apoptosis of NSCLC cells, were assessed. The relationship between TAOK1 and WW and C2 domain containing 1 (WWC1) was assessed by Co-IP assay. The subcutaneous injection of tumor cells in nude mice was used to verify it in vivo.

**Results:**

As expected, TAOK1 was increased in NSCLC cell lines. Following TAOK1 knockdown, NSCLC cells exhibited a significant decrease in the invasion and increased apoptosis in vitro. Instead, the TAOK1 elevation showed the opposite results. The Co-IP assay identified that TAOK1 specifically interacted with WWC1. Knockdown of WWC1 overturned TAOK1 silencing-mediated malignant phenotype of NSCLC cells. Additionally, subcutaneous tumorigenesis assays in nude mice confirmed that TAOK1 knockdown markedly restrained the proliferation capacity of NSCLC cells in vivo.

**Conclusion:**

Surprisingly, TAOK1 overexpression in NSCLC promotes tumor cell growth and invasion, which is associated with downregulation of its downstream protein WWC1, and this result might provide a robust research basis to inquire about the precise therapeutic targets for NSCLC.

## 1. Introduction

Despite increasing awareness and attention to physical health, lung cancer incidence is still rising. Lung cancer accounts for 13% of all cancer cases worldwide and 23% of all cancer-related deaths in 2018 worldwide [1]. According to the lung cancer classification guidelines published by the World Health Organization in 2015, lung cancer is divided into small cell lung cancer and non-small-cell lung cancer (NSCLC), which the latter accounts for more than 80% of the total incidence of lung cancer but are more abundant than the latter treatment. Due to the insidious early symptoms of lung cancer, some patients are already advanced or locally advanced at the time of diagnosis, leading to poor treatment outcomes and poor prognosis [2]. Surgical resection contributes to NSCLC patients' long-term survival, and chemoradiotherapy is therapeutic for patients with advanced disease [3]. Consequently, it is urgent to explore NSCLC pathogenesis and new treatments.

Thousand and one amino-acid protein kinases (TAOKs) consist of three members, including TAOK1, TAOK2, and TAOK3. They are part of the step 20p protein kinase family, which plays essential roles upstream in the mitogen-activated protein kinase cascade, thus participating in multiple cellular processes [4]. TAOK1, also known as PSK2, TAO1, or MARKK, participates in apoptotic morphology through c-Jun N-terminal and Rho kinase-1 [5]. Draviam et al. reported that the interaction between TAOK1 and components of the spindle checkpoint is widely involved in mitotic progression [6]. A previous study indicated that TAOK1 is essential in neuronal function, involved in neurite outgrowth and axonal transport, and the differentiation of PC12 cells [7]. Li et al. found that TAOK1 reduces the release of inflammatory factors and the antiapoptotic ability in rats subjected to MCAO by regulating the PI3K/AKT and MAPK pathways, playing a protective role in cerebral ischemic stroke [8]. In the experimental model of inflammatory bowel disease, TAOK1 markedly suppresses colitis by downregulating the formation of the IL-17RA and Act1 complex [9]. According to a substantial study, TAOK1 was a downstream target for miRNA-706, and miRNA-706 inhibited hepatic fibrogenesis by downregulating TAOK1 [10]. Furthermore, current evidence demonstrated that the dysregulation of the Ste20 kinase pathway is closely related to malignant tumors, and TAOK1 inhibitors arrested NSCLC cells in G0/G1 phase and induced cell apoptosis, which indicates TAOK1 might play a crucial role in the pathogenesis of lung cancer [11]. Currently, studies targeting toak1 in NSCLC are in their infancy, and its pathophysiological functions need to be further mined.

WWC1, also known as KIBRA, is characterized by two WW domains in the amino terminus, an internal C2-like domain and a carboxy-terminal glutamic acid-rich stretch [12]. As a well-known tumor suppressor gene in various cancer, WWC1 participates in the regulation of cell proliferation, differentiation, and metastasis. However, the effect of TAOK1 on WWC1 in NSCLC progression and the potential mechanism remains unknown.

In the present study, we indicate that TAOK1 expression is upregulated in NSCLC cell lines. Functional studies showed that TAOK1 regulates NSCLC cell behavior and tumor formation in vivo. Mechanistic investigations suggest that TAOK1 interacts with WWC1 and regulates WWC1 expression, thereby promoting NSCLC progression.

## 2. Materials and Methods

### 2.1. Cell Culture and Transfection

Shanghai Cell Bank provided the NSCLC cell lines (H1650, PG49, H1299, and A549) and the normal bronchial epithelial cell line BEAS-2B. All cells were supplemented with appropriate concentrations of serum, for which BEAS-2B and A549 cells were cultured in DMEM containing 10% FBS; H1650, PG49, and 1299 cells were maintained in RPMI 1640 medium at 37°C in 5% CO_2_. To keep the cells growing well, NSCLC cells were seeded in 6-well plates and cultured for 24 h. Short-hairpin RNA (shRNA) (sh-TAOK1), negative control (sh-NC), TAOK1 overexpression plasmid by pcDNA3.1 vector (pcDNA3.1-TAOK1), and negative control (pcDNA3.1-NC) (Thermo Fisher Scientific, Waltham, MA, USA) were transfected into the target cells using Lipofectamine 2000 transfection reagent (Invitrogen).

### 2.2. Quantitative Real-Time Polymerase Chain Reaction (qRT-PCR)

Total RNA was extracted from NSCLC cells according to the TRIzol reagent instructions, reverse transcribed into cDNA according to the instructions of the reverse transcription kit (Promega, USA), and then amplified using cDNA as a template, and *β*-actin was used as an internal reference for qRT-PCR amplification. The relative gene expression was calculated using the 2^−*ΔΔ*Ct^ method. Primer sequences were as follows: GAPDH F: 5′-CCTCGTCTCATAGACAAGATGGT-3′, R: 5′-GGGTAGAGTCATACTGGAACATG-3′; TAOK1 F: 5′-AAG AGC ATC AGC TCC ACA GT-3′, R: 5′-GCC GAT GTT CGT CCA TTT CT-3′; and WWC1 F: 5′-TCCGCAGTCCTGGAAACATT-3′ (forward), R: 5′-GTGGATTCCCAATGAGCCGA-3′.

### 2.3. Western Blotting

Transfected NSCLC cells were charged, and the supernatant was collected to examine the protein concentration after adding the RIPA lysis buffer. Subsequently, electrophoretic samples were configured and added to 10% SDS-PAGE gels for electrophoresis experiments. The proteins on the gels were then transferred to PVDF membranes and blocked with 5% nonfat milk for at least 2 h. Primary antibodies (TAOK1 and WWC1) were added to the membranes and incubated for 12-16 h at 4°C, after which the membranes were washed three times for 10 min each with TTBS. The corresponding rabbit/mouse secondary antibodies were added and incubated for 2 h at room temperature, after which the membranes were rewashed three times for 10 min each. Finally, ECL reagents were used to evaluate the grayscale of each band quantitatively.

### 2.4. Cell Counting Kit-8 (CCK-8) Assay

Logarithmic growth phase NSCLC cells were taken, the cell suspension was prepared, and the cells (1 × 10^4^ cells/well) were seeded in 96-well plates and grew in a 5% CO_2_ incubator for 24, 48, and 72 h, respectively. Next, 10 *μ*L of CCK-8 solution was added 2 h before each assay time point and placed plates in the incubator for 1 h, then placed into a microplate reader to detect absorbance values at a wavelength of 450 nm.

### 2.5. Ethynyl Deoxyuridine (EdU) Incorporation Assay

NSCLC cells (1 × 10^4^ cells/well) were plated in 96-well plates. After overnight incubation, 1 : 1000 dilution of EDU reagent was added, cells were washed with PBS after 2 h incubation and then fixed with 3% paraformaldehyde for 10 min. Afterward, 2 mg/mL glycine was added for 5 min incubation. 0.5% Triton X-100 was added for 10 min. Apollo staining solution was added after washing and incubated for 30 min in the dark. Nuclei were then stained with Hoechst for 10 min. After washing, count the analysis after taking photographs under a microscope.

### 2.6. Flow Cytometry

100 *μ*L of binding buffer was utilized to resuspend NSCLC cells. After adding 5 *μ*L Annexin V-FITC in cells for 15 min in the dark at room temperature, the PI solution was remixed. The apoptosis rate of each group was measured by flow cytometry.

### 2.7. Transwell Cell Invasion Assay

Transwell chambers were purchased from Corning with a pore size of 8.0. NSCLC cells were digested and prepared into cell suspension, counted, and the concentration was adjusted to 2 × l0^5^/mL and seeded in the upper chamber with coated Matrigel. Meanwhile, a complete medium was put into the lower chamber of the culture plate. Further, cells with 4% paraformaldehyde and methanol were added to the culture plate to, respectively, fixed for 20 min, and gentian violet was added to stain for 15 min. Clean the chamber upper chamber with PBS, and carefully wipe the cells on the membrane surface at the bottom of the upper chamber with a wet cotton swab. After drying the chamber upper chamber, count and take photos with the burning inverted microscope.

### 2.8. Co-Immunoprecipitation (Co-IP)

NSCLC cells are lysed in lysis buffer to obtain cell lysate, followed by incubated with agarose bead-conjugated antibodies against anti-TAOK1 and anti-WWC1 overnight. Further, the beads were washed to harvest the binding proteins. Finally, western blotting was used to assess immunoprecipitated protein.

### 2.9. Immunohistochemistry (IHC)

Surgically resected tumor tissues were fixed in 10% formalin and processed for embedding, whereas tissue sections were made with a slice thickness of 4 *μ*M. Sections were deparaffinized in xylene, rehydrated, heat-fixed in sodium citrate (pH 6.0) buffer, blocked in 3% hydrogen peroxide, and incubated with a rabbit polyclonal antibody against Ki-67 at a concentration of 1 : 200 at 4°C for 18 h. The next day, secondary antibodies for histochemistry were added to the sections, stained with DAB, and counterstained with Mayer's hematoxylin. Sections were observed and photographed with a microscope (Nikon).

### 2.10. Tumor Xenograft Assay

24 male BALB/c nude mice (four weeks old) were brought from Cavens Laboratory Animals Co., Ltd. (Changzhou, China). TAOK1 targeting shRNA (sh-TAOK1) or scrambled shRNA were transfected into A549 cells, followed by subcutaneous injection into the flanks of the nude mice at a density of 5 × 10^6^ cells. Tumor volume was assessed by measuring tumor diameters every week.

### 2.11. PPI Network Construction

The PPI network was carried out using the Search Tool for the Retrieval of Interacting Genes and proteins (STRING) database (ver. 10.0, http://www.string-db.org/). The network visualization software Cytoscape was applied to create the PPI interaction network.

### 2.12. Statistical Analysis

Statistical analysis of experimental data was processed using SPSS 23.0 (SPSS Inc., Chicago, IL). Data were expressed as mean ± SD. The significance of the variance between the two groups was determined by Student's *t*-test. *P* < 0.05 was considered statistically significant.

## 3. Results

### 3.1. TAOK1 Was Found to Be Increased in NSCLC Cell Lines

To examine the role of TAOK1 in CC, the expression of TAOK1 was evaluated in NSCLC cell lines by western blotting. It is worth noting that TAOK1 was highly expressed in H1650, PG49, H1299, and A549 cells compared to the normal lung cell line (BEAS-2B) (Figure 1(a)).

### 3.2. TAOK1 Knockdown Reduced Proliferation, Migration, and Antiapoptotic Ability of NSCLC Cells

To explore the biological function of TAOK1, we constructed TAOK1 stably silenced H1299 and A549 cells, respectively. Western blot assay showed that TAOK1 interference effectively enhanced TAOK1 expression levels in H1299 and A549 cells (Figure 2(a)). After silencing TAOK1, the proliferation ability of H1299 and A549 cells was decreased (Figure 2(b)). We also found that cell proliferation was remarkably suppressed in TAOK1-depleted H1299 and A549 cells using the EdU assay (Figure 2(c)). Transwell assay demonstrated that TAOK1 knockdown significantly reduced the number of invading H1299 and A549 cells (Figure 2(d)). Besides, flow cytometry results indicated that TAOK1 knockdown significantly induced apoptosis (Figure 2(e)).

### 3.3. TAOK1 Overexpression Promoted Proliferation, Invasion, and Reduced Apoptosis of NSCLC Cells

We next elevated TAOK1 expression into H1299 and A549 cells. Using western blotting, we found that the introduction of pcDNA-TAOK1 caused an efficient increase in TAOK1 protein levels (Figure 3(a)). Compared with the pcDNA group, TAOK1 overexpression conspicuously promoted both A549 and NCI-H1299 cell proliferation (Figure 3(b)). EdU assay also revealed that TAOK1 overexpression facilitated A549 and NCI-H1299 cell growth (Figure 3(c)). Transwell assay demonstrated that the number of invaded cells elevated after TAOK1 overexpressing (Figure 3(d)). We also observed a significant decrease in apoptosis in TAOK1 overexpressing A549 and H1299 cells (Figure 3(e)).

### 3.4. TAOK1 Bound with WWC1 and Negatively Regulated WWC1 Expression

Given the impact of TAOK1 in NSCLC cell behavior, we performed a STRING interaction network analysis of TAOK1 and its associated significantly differentially expressed genes. The result demonstrated a potential binding relationship between TAOK1 and WWC1 proteins (Figure 4(a)). Subsequently, we investigated the interaction between TAOK1 and WWC1 by co-immunoprecipitation (Co-IP) assay. The results indicated that compared with control IgG, TAOK1-antibody could pull down WWC1. Correspondingly, WWC1-antibody also pulled down TAOK1 (Figures 4(b) and 4(c)), which indicated that TAOK1 could be intact with WWC1 in A549 cells. Besides, western blotting revealed that the TAOK1 interference restrained the WWC1 protein level in A549 cells, whereas overexpression of TAOK1 led to opposite results (Figure 4(d)).

### 3.5. WWC1 Knockdown Reversed TAOK1 Knockdown-Mediated Effect on Proliferation, Invasion, and Apoptosis of NSCLC Cells

To further investigate whether TAOK1 affects the NSCLC cellular fates through WWC1, TAOK1 shRNA alone, or WWC1 shRNA were transfected into A549 and H1299 cells. Western blotting results uncovered that WWC1 interference overturned the facilitation effect of TAOK1 interference on WWC1 expression (Figure 5(a)). From the results of CCK-8, we confirmed that the capacity of cell proliferation was reduced by silencing TAOK1, whereas it was restored byWWC1 knockdown (Figure 5(b)). EdU assay also revealed that shTAOK1 inhibited A549 and NCI-H1299 cell growth (Figure 5(c)). As expected, Transwell and flow cytometry assays also indicated that TAOK1 silencing inhibited cell invasion and antiapoptosis abilities, whereas WWC1 knockdown could invert these changes (Figures 5(d) and 5(e)).

### 3.6. TAOK1 Knockdown Suppressed Xenograft Tumor Growth in Mice

To further detect whether TAOK1 silencing could inhibit tumor growth, A549 cells transfected with TAOK1 shRNA were subcutaneously injected into nude mice. TAOK1 knockdown significantly repressed tumor growth, reducing tumor volume and weight (Figures 6(a)–6(c)). Western blotting results revealed that TAOK1 silencing decreased TAOK1 protein expression and increased WWC1 levels in tumor tissues of rats (Figures 6(d) and 6(e)). Additionally, the immunohistochemistry assay showed that TAOK1 interference significantly attenuated the Ki-67 expression level (Figure 6(f)).

## 4. Discussion

The acquisition of the function of some oncogenes and the loss of the function of many tumor suppressor genes are the central links between tumor genesis and initiation. TAOK1 belongs to the mammalian STE20 kinase family, and its alteration, in turn, leads to changes in the biological behavior of cells, allowing uncontrolled cancer cell growth, aberrant proliferation, transformation and motility, and ultimately invasion and metastasis [13, 14]. Gao et al. indicated that TAOK1 inhibition or depletion effectively inhibits cell growth by arresting cell mitosis [15]. It was reported that TAOK1 expression was prominently reduced in HCC tissues and was positively correlated with immune infiltration in HCC [16]. Shi et al. validated that TAOK1 is a direct target of miR-706 cells accountable for EMT in hepatic fibrosis [16]. Meanwhile, overexpression of TAOK1 was uncovered in colorectal cancer tissues [17]. Moreover, serine/threonine kinase expression in cancers was investigated by in situ hybridization. The results suggested that increased expression of TAOK1 in lung cancer tissues showed high levels relative to lung tissues [17]. Evidence has revealed that TAOK1 might function as a Hippo pathway gene and is the main element of the susceptibility of lung cancer cells [18]. Given the above literature, an in-depth study of TAOK1 molecular expression in NSCLC and the effect of altered TAOK1 molecular expression levels on the biological behavior of NSCLC cells is essential to gain insight into the mechanism of NSCLC development and progression. Here, we uncovered that TAOK1 was upregulated in NSCLC cell lines. Subsequent functional studies revealed that knockdown of TAOK1 efficiently inhibited NSCLC cell proliferation, invasion, and induced apoptosis in vitro and suppressed NSCLC xenograft growth in vivo. Conversely, overexpression of TAOK1 promoted NSCLC cell proliferation and invasion and inhibited apoptosis.

A previous study has demonstrated that breast cancer patients with low expression WWC1 genes usually have larger tumor sizes and poor prognoses [19]. A previous study revealed that WWC1 overexpression hindered the SOX2-induced migration ability and invasive potential in esophageal squamous cell carcinoma [20]. WWC1 was low expressed in colorectal cancer tissues, and low-level WWC1 indicated worse survival of colorectal cancer patients [21]. Most importantly, WWC1 was one of the well-known upstream regulators of the Hippo signaling pathway, which contributes to the activation of the Hippo signaling pathway, resulting in YAP phosphorylation [22]. Another study has revealed that WWC1 cooperated with NF2 to mitigate the malignant progression of intrahepatic cholangiocarcinoma by activation of LATS1/2 and inhibition of YAP/TAZ activity [23]. It was reported that WWC1 was downregulated in lung adenocarcinoma tissues and cells, and WWC1 restrained proliferation and invasion and accelerated apoptosis of lung adenocarcinoma cells by Hippo signaling pathway [24]. Moreover, ACTL6A contributed to tumorigenesis in vitro and in vivo by silencing WWC1 expression and regulating Hippo/YAP signaling [25]. This study showed that TAOK1 interacted with WWC1 and negatively regulated WWC1 expression. Intriguingly, WWC1 interference restored the effects of TAOK1 knockdown on NSCLC cell proliferation, invasion, and apoptosis. However, this study still has some limitations, and it would be better to add some more animal experiments. This study lacks related clinical research, and it still needs to be further validated in a larger patient cohort.

In conclusion, our study identified that TAOK1 was low expressed in NSCLC cell lines. Furthermore, TAOK1 contributed to tumor-promoting effects, manifested by facilitating NSCLC cell proliferation, invasion, and suppressing apoptosis in vitro and accelerating xenograft formation in vivo by reducing WWC1 expression. The above findings provide a theoretical understanding of the oncogenic mechanisms of TAOK1 in NSCLC and a potential candidate for the therapy of NSCLC.

## Figures and Tables

**Figure 1:** TAOK1 was highly expressed in NSCLC cell lines. (a, b) Relative TAOK1 expression in human NSCLC cell lines (H1650, PG49, H1299, and A549) and the normal lung cell line (BEAS-2B). ^∗^*P* < 0.05.

**Figure 2:** Effects of TAOK1 silencing on NSCLC cell biological behavior. A549 and H1299 cells were transfected with TAOK1 shRNA and corresponding negative controls, respectively. (a) Western blotting analysis of TAOK1 levels. (b–e) The proliferation, invasion, and antiapoptosis ability of TAOK1 silenced and control cells were detected by CCK-8, EdU, Transwell, and flow cytometry assays, respectively. ^∗^*P* < 0.05.

**Figure 3:** Effects of TAOK1 overexpression on NSCLC cell biological behavior. A549 and H1299 cells were transfected with pcDNA-TAOK1 and corresponding negative controls, respectively. (a) Western blotting analysis of TAOK1 levels. (b–e) The proliferation, invasion, and antiapoptosis ability of TAOK1 elevated and control cells were detected by CCK-8, EDU, Transwell, and flow cytometry assays, respectively. ^∗^*P* < 0.05.

**Figure 4:** TAOK1 interacted with WWC1 and inhibited WWC1 expression. (a) Interaction network analysis diagram of TAOK1. (b, c) Co-IP assay analysis of TAOK1 and WWC1 binding. (d) Western blotting analysis of WWC1 levels. ^∗^*P* < 0.05.

**Figure 5:** WWC1 knockdown reversed the function of TAOK1 on NSCLC cell biological behavior. A549 and H1299 cells were transfected with sh-TAOK1 alone or together with sh-WWC1. (a) Western blotting analysis of TAOK1 levels. (b–e) The proliferation, invasion, and antiapoptosis ability of TAOK1 silenced, and concurrently WWC1 silenced, and control cells were detected by CCK-8, EdU, Transwell, and flow cytometry assays, respectively. ^∗^*P* < 0.05.

**Figure 6:** TAOK1 interference restrained tumor development in vivo. (a) The images of tumors in each group. (b, c) The volume and weight of tumor in each group. (d) Relative TAOK1 and WWC1 expression in tumor tissues in each group. (e) Immunohistochemistry analysis of each group's relative Ki-67 protein levels in tumor tissues. ^∗^*P* < 0.05.

## Data Availability

The labeled dataset used to support the findings of this study are available from the corresponding author upon request.
